The article "Integrated Lipidomics in the Secreted Phospholipase A2 Biology" was published in 2011. Journal: Int J Mol Sci.

# Integrated Lipidomics in the Secreted Phospholipase A_2_ Biology

**DOI:** 10.3390/ijms12031474

**Published:** 2011-02-25

**Authors:** Makoto Murakami, Hiroyasu Sato, Yoshitaka Taketomi, Kei Yamamoto

**Affiliations:** Lipid Metabolism Project, The Tokyo Metropolitan Institute of Medical Science, 2-1-6 Kamikitazawa, Setagaya-ku, Tokyo 156-8506, Japan; E-Mails: sato-hr@igakuken.or.jp (H.S.); taketomi-ys@igakuken.or.jp (Y.T.); and yamamoto-ki@igakuken.or.jp (K.Y.)

**Keywords:** phospholipase A_2_, phospholipid, lipidomics, transgenic mouse, knockout mouse

## Abstract

Mammalian genomes encode genes for more than 30 phospholipase A_2_s (PLA_2_s) or related enzymes, which are subdivided into several subgroups based on their structures, catalytic mechanisms, localizations and evolutionary relationships. More than one third of the PLA_2_ enzymes belong to the secreted PLA_2_ (sPLA_2_) family, which consists of low-molecular-weight, Ca^2+^-requiring extracellular enzymes, with a His-Asp catalytic dyad. Individual sPLA_2_ isoforms exhibit unique tissue and cellular localizations and enzymatic properties, suggesting their distinct pathophysiological roles. Recent studies using transgenic and knockout mice for several sPLA_2_ isoforms, in combination with lipidomics approaches, have revealed their distinct contributions to various biological events. Herein, we will describe several examples of sPLA_2_-mediated phospholipid metabolism *in vivo,* as revealed by integrated analysis of sPLA_2_ transgenic/knockout mice and lipid mass spectrometry. Knowledge obtained from this approach greatly contributes to expanding our understanding of the sPLA_2_ biology and pathophysiology.

## 1. Introduction

Phospholipase A_2_ (PLA_2_) hydrolyzes the *sn*-2 position of glycerophospholipids to yield fatty acids and lysophospholipids. In the view of signal transduction, the PLA_2_ reaction has been considered to be of particular importance since arachidonic acid, one of the polyunsaturated fatty acids (PUFAs) released by PLA_2_, is metabolized to various lipid mediators such as prostaglandins and leukotrienes. In addition, lysophospholipids or its metabolites, such as lysophosphatidic acid and platelet-activating factor, also represent another class of lipid mediators. These lipid mediators exert numerous biological actions through their cognate G protein-coupled receptors on target cells. PLA_2_ has also been implicated in membrane glycerophospholipid remodeling, thereby contributing to cellular homeostasis.

Mammalian genomes encode more than 30 PLA_2_s or related enzymes, which are classified into several subgroups on the basis of their primary structures and functions. Critical contributions of the intracellular PLA_2_ families, namely cytosolic PLA_2_s (cPLA_2_s) and Ca^2+^-independent PLA_2_s (iPLA_2_s), to aracidnonic acid metabolism and membrane homeostasis, respectively, have been well established by numerous studies [1,2]. The secreted PLA_2_ (sPLA_2_) family represents structurally related, disulfide-rich, low molecular weight, lipolytic enzymes with a His-Asp catalytic dyad. sPLA_2_s occur in a wide variety of vertebrate and invertebrate animals, plants, fungus, bacteria, and viruses, and 11 sPLA_2_ isozymes (IB, IIA, IIC, IID, IIE, IIF, III, V, X, XIIA and XIIB) have been identified in mammals [2–4]. Of these, sPLA_2_s belonging to the group I/II/V/X collection (conventional sPLA_2_s) are closely related, 14–19-kDa secreted enzymes with a highly conserved Ca^2+^-binding loop (XCGXGG) and a catalytic site (DXCCXXHD). In addition to these elements, there are six absolutely conserved disulfide bonds and up to two additional unique disulfide bonds, which contribute to the high degree of stability of these enzymes. Group III and group XII sPLA_2_s (atypical sPLA_2_s) share homology with the I/II/V/X collection of sPLA_2_s only in the Ca^2+^-binding loop and catalytic site, thereby representing the group III and XII collections, respectively. sPLA_2_ enzymes hydrolyze the ester bond at the *sn*-2 position of glycerophospholipids with distinct selectivity toward *sn*-2 fatty acids and polar head groups in the presence of mM concentrations of Ca^2+^. Since individual sPLA_2_s display distinct cellular/tissue distributions and substrate head group specificities, they may play non-redundant, isoform-specific roles *in vivo*.

Although many potential functions of sPLA_2_s have been proposed on the basis of *in vitro* studies, the precise biological roles and relevant target membranes of these enzymes *in vivo* have remained elusive until recently. Several, if not all, sPLA_2_s are capable of releasing arachidonic acid from cultured cell membranes when overexpressed or added exogenously at excess amounts *in vitro* [2–4]. However, it still remains controversial whether this function could indeed be operated by sPLA_2_s *in vivo*. The reason why sPLA_2_s are secreted is most probably because sPLA_2_s participate in pathophysiology by regulating *extracellular* phospholipid metabolism, which include adjacent cell membranes (plasma membranes or microvesicles shed from cells), non-cellular lipid components such as lipoproteins and pulmonary surfactant, and foreign phospholipids such as microbe membranes and dietary lipids. The *in vitro* actions of individual sPLA_2_s on various target membranes are summarized in Table 1. This target variation may explain the molecular evolution of a number of sPLA_2_s with distinct localizations and substrate specificities. Therefore, once some phenotypes appear in sPLA_2_-knockout or -transgenic mice, this could be attributable to a combination of these varied actions rather than only by alterations in lipid mediator levels.

In the past few years, we have analyzed the phenotypes of transgenic or knockout mice for several sPLA_2_ isozymes, in combination with a lipid profiling technique by mass spectrometry. This integrated approach, together with studies using these mice by other research groups, has helped us understand the potential action of a given sPLA_2_ on particular target membranes and its impact on pathophysiology *in vivo*. In this article, we will give an overview of current analyses on transgenic or knockout mice for two particular conventional sPLA_2_s, group V and X, and an atypical sPLA_2_, group III. Also, we will give a brief summary of pathophysiological functions of other sPLA_2_s that have been clarified to date.

## 2. Biological Functions of sPLA_2_s *in Vivo*

### 2.1. Group V sPLA_2_ (sPLA_2_-V)

Among the conventional sPLA_2_s, sPLA_2_-V has the simplest structure. It lacks group I- and II-specific disulfide bonds, group II-specific C-terminal extension, and group I- or X-specific N-terminal propeptide [5]. However, sPLA_2_-V is evolutionally close to group II sPLA_2_s, since the *Pla2g5* gene resides within the gene cluster for the group II subfamily of sPLA_2_s. sPLA_2_-V is expressed at the highest level in the heart, followed by the lung. In the lung, sPLA_2_-V is expressed in the airway epithelium and alveolar macrophages, and its expression is markedly elevated in mice receiving models of asthma or acute respiratory distress syndrome (ARDS) [6]. Immunohistochemistry and *in situ* hybridization of sPLA_2_-V clearly indicate its location in the bronchial epithelium of patients with severe pneumonia [7].

To assess the biological functions of sPLA_2_-V, we generated transgenic mice overexpressing this enzyme in the whole body (*Pla2g5*-Tg) [8]. We found that *Pla2g5*-Tg mice died in the neonatal period (within 8 h after birth) due to respiratory failure. The lungs of *Pla2g5*-Tg mice exhibited atelectasis with thickened alveolar walls and narrow air spaces, accompanied by infiltration of macrophages and only modest elevations in eicosanoid levels. This severe pulmonary defect in *Pla2g5*-Tg mice was attributable to marked reduction of the lung surfactant phospholipids, phosphatidylcholine (PC) (Figure 1a) and phosphatidylglycerol (PG) (Figure 1b), as demonstrated by ESI-MS (electrospray ionization mass spectrometry) analysis.

The principal function of lung surfactant, which is a mixture of phospholipids (90%) and surfactant proteins (10%), is to reduce the work of breathing by lowering alveolar surface tension during respiration. PC with saturated and monosaturated fatty acids (palmitic acid in particular) is predominant in surfactant phospholipids (∼80% of total lipid) [9], and PG (∼10% of total lipid) plays a role in phospholipid-protein interactions that maintain the alveolar surfactant layer, especially through interaction with the surfactant protein SP-B [10]. Since changes in the ratio of the surfactant components can dramatically alter the surface tension in small airways and alveoli, compromising airway patency, gas exchange and host defense, any surfactant abnormality can have severe pathological consequences in terms of lung function. Indeed, previous studies have indicated a role of sPLA_2_s in inflammation-mediated surfactant malfunction through hydrolysis of surfactant phospholipids [11–18]. Aberrant hydrolysis of surfactant phospholipids leads to ARDS, which is a clinically and pathologically complex syndrome due to acute life-threatening lung injury involving an alteration of pulmonary surfactant, and numerous predisposing factors can be involved in the etiology, including pneumonia and sepsis [9]. Hydrolysis of surfactant phospholipids is an early pathological event of ARDS, and hydrolysis of as little as 10–15% of surfactant can cause this serious condition. Levels of sPLA_2_ activity in bronchoalveolar fluid (BALF) of patients with ARDS are often positively correlated with disease severity [11–14], and chemical sPLA_2_ inhibitors that block classical sPLA_2_s protect animals against experimental ARDS or related lung injury [15]. Given that the expression of sPLA_2_-V is greatly elevated in human lungs with severe inflammation [7] and in cultured human bronchial epithelial cells stimulated with pro-inflammatory cytokines (Figure 1c), that sPLA_2_-V can efficiently hydrolyze lung surfactant phospholipids *in vitro* [16,18], and that the neonatal death of *Pla2g5*-Tg mice is in many aspects similar to that observed in mutant mice manipulated for a panel of genes that have been implicated in surfactant homeostasis [19,20], sPLA_2_-V may contribute to ongoing surfactant hydrolysis often observed in the lungs of patients with ARDS (Figure 1d).

Following our study using *Pla2g5*-Tg mice as shown above, three studies using mice null for sPLA_2_-V (*Pla2g5^−/−^*) by other groups have delineated the crucial contribution of this sPLA_2_ isoform to mouse airway disease models [6,21,22]. Thus, the allergen (ovalbumin or house dust mite)-induced, Th2-dependent asthmatic models, as well as the LPS-induced ARDS model, were significantly reduced in *Pla2g5^−/−^* mice compared with replicate *Pla2g5^+/+^* mice [6,21]. In the asthmatic models, the action of sPLA_2_-V occurs in two regulatory steps; one at the step of antigen uptake and processing by dendritic cells leading to the initiation of the Th2 response, and the other at the step of airway-resident cells which may contribute to the propagation of airway inflammation [22]. The airway-resident cell-dependent pathway requires catalytic activity of sPLA_2_-V, since aerosolized intake of native, but not mutant, sPLA_2_-V caused a dose-related increase of airway resistance, persistent airway narrowing, and leukocyte migration, and since intratracheal application of a neutralizing antibody against sPLA_2_-V ameliorated the asthmatic response [6]. However, eicosanoid levels in BALF were unchanged in this model, suggesting that the airway action of sPLA_2_-V does not profoundly depend on lipid mediators. Although the molecular mechanism underlying the airway-resident cell-dependent pathway has not yet been clarified, we speculate that the protection from disease-associated surfactant hydrolysis by the absence of sPLA_2_-V may be a likely explanation for this event. Thus, blockade of endogenous sPLA_2_-V could provide a potential new therapeutic approach for treating diverse phenotypes of human asthma.

Studies using *Pla2g5^−/−^* mice have also revealed unique functions of sPLA_2_-V in inflammation, host defense, and atherosclerosis. *Pla2g5^−/−^* mice displayed reduced zymosan-induced peritonitis since peritoneal macrophages produced less eicosanoids [23], were protected from *Candida albicans* infection since phagocytic killing of the fungi by macrophage was reduced [24,25], and were more sensitive to inflammatory arthritis since phagocytosis of the pro-inflammatory immune-complex by macrophages was reduced in the joints [26]. sPLA_2_-V can also potently hydrolyze phospholipids in low-density (LDL) and high-density (HDL) lipoprotein particles, and LDL receptor-deficient mice transplanted with *Pla2g5^−/−^* bone marrow cells are partially protected from atherosclerosis development [27]. Furthermore, a recent single nucleotide polymorphism analysis has revealed an association of the human sPLA_2_-V gene haplotype with plasma LDL levels in patients with type 2 diabetes [28], suggesting its metabolic role.

### 2.2. Group X sPLA_2_ (sPLA_2_-X)

Structurally, sPLA_2_-X has both the group I- and II-specific properties. Unlike sPLA_2_-V, which is constitutively active once synthesized, sPLA_2_-X is synthesized as an inactive zymogen and converted to an active enzyme by proteolytic removal of the N-terminal propeptide [29]. Amongst the sPLA_2_ members, sPLA_2_-X shows the highest affinity for PC and thereby for the PC-rich outer leaflet in the plasma membrane of mammalian cells [30,31]. Accordingly, supplementation or forcible transfection of exogenous sPLA_2_-X results in increased release of arachidonic acid and its oxygenated metabolites in many cell types. However, these results should be carefully interpreted, because unlike cPLA_2_α, which is ubiquitously expressed and is a central player of arachidonic acid release [1], the expression of sPLA_2_-X is tissue- or cell-specific. In fact, sPLA_2_-X is constitutively expressed at high levels in the genital and digestive organs, where they play roles in sperm activation and gastrointestinal phospholipid digestion, respectively, independently of lipid mediator production [32,33].

In the lung, sPLA_2_-X is focally expressed in airway epithelial cells, and its expression is elevated in the epithelium as well as in alveolar macrophages following asthmatic challenge in both mice and humans [34,35]. The contribution of sPLA_2_-X to airway inflammation was confirmed by a study using mice lacking this enzyme (*Pla2g10^−/−^*), in which the ovalbumin-induced, Th2-dependent asthmatic responses in the airway, including infiltrations of CD4^+^ and CD8^+^ T cells and eosinophils, mucus secretion, elevation of Th2 cytokines, and production of pro-asthmatic lipid mediators such as cysteinyl leukotrienes and prostaglandin D_2_ (PGD_2_), were markedly reduced [34]. Taken together with the evidence from *Pla2g5^−/−^* mice (see above), it has become obvious that the two particular sPLA_2_s, sPLA_2_-V and -X, participate in the asthma pathology. In addition, *Pla2g10^−/−^* mice are protected from neutrophil-induced myocardial damage following ischemia-reperfusion, where sPLA_2_-X is involved in the production of leukotriene B_4_ (LTB_4_) by neutrophils [36].

In order to address the *in vivo* action of sPLA_2_-X, we produced transgenic mice overexpressing this enzyme in the whole body (*Pla2g10*-Tg) [8]. Unexpectedly, in contrast to *Pla2g5*-Tg neonates that exhibited fatal respiratory failure (see above), systemic *Pla2g10*-Tg mice displayed no apparent abnormality of the respiratory tract with normal alveolar architecture and surfactant composition [8], despite the fact that sPLA_2_-X can potently hydrolyze surfactant PC *in vitro* [18]. This surprising result turned out to be because sPLA_2_-X protein existed as an inactive zymogen in most tissues. The active form of sPLA_2_-X was produced at inflamed sites in *Pla2g10*-Tg mice [8]. These results suggest that sPLA_2_-X mostly exists as an inactive zymogen under physiological conditions and that its proteolytic activation occurs during inflammation. In contrast, macrophage-specific *Pla2g10*-Tg mice developed severe lung inflammation which led to early death by 2∼3-weeks of age [37]. Although the discrepancy between systemic and macrophage-specific *Pla2g10*-Tg mice is unclear, sPLA_2_-X expressed in alveolar macrophages might be efficiently converted by proteolytic processing to an active form.

Although systemic *Pla2g10*-Tg mice did not have any alveolar injury, we found a remarkable phenotype in these mice before weaning: they developed alopecia [38]. Although pelage hairs of *Pla2g10*-Tg mice initially grew, complete but transient hair loss was observed at 3–4 weeks of age, a period corresponding to the late stage of the initial hair cycle (Figure 2a). Proteolytic activation of sPLA_2_-X in *Pla2g10*-Tg skin temporally preceded hair loss. Histological analyses of the alopecic *Pla2g10*-Tg skin revealed hair follicle distortion, hyperkeratosis and sebaceous gland hyperplasia (Figure 2b), which were accompanied by increased expression of genes related to terminal differentiation of epidermis and reduced expression of genes related to hair development. ESI-MS analysis of *Pla2g10*-Tg skin revealed that sPLA_2_-X hydrolyzed phosphatidylethanolamine (PE), but not PC, molecular species to yield PUFAs (Figure 2c), which were further converted to some if not all eicosanoids. A schematic model for the action of sPLA_2_-X in *Pla2g10*-Tg skin is illustrated in Figure 2d. These results, together with the finding that endogenous sPLA_2_-X shows a hair cycle-dependent periodic expression in the outer root sheath of hair follicles in mouse skin (Figure 2e) [38], suggest a potential functional link between sPLA_2_-X and skin biology, and may provide a molecular explanation for the skin abnormality induced by aberrant expression of other sPLA_2_s such as sPLA_2_-IIA, whose transgenic mice also developed alopecia [39]. Importantly, in *Pla2g10^−/−^* mice, hair growth in the anagen phase was significantly delayed, and this was caused by growth retardation of the outer root sheath in hair follicles [40]. Thus, sPLA_2_-X intrinsically functions in the hair quality control.

The ability of sPLA_2_-X to potently hydrolyze phospholipids in LDL and HDL *in vitro* has led to the hypothesis that, as in the case of sPLA_2_-V (see above), sPLA_2_-X may also participate in atherosclerosis. Indeed, sPLA_2_-X-hydrolyzed LDL particles promote foam cell formation from mouse peritoneal macrophages [41]. These *in vitro* observations may be relevant to cardiovascular pathology, since *Pla2g10^−/−^* mice are protected from angiotensin-II-induced aortic aneurysm and atherosclerosis [42]. sPLA_2_-X-released PUFAs negatively regulates liver X receptor (LXR), and accordingly, deficiency of sPLA_2_-X results in augmented LXR activation leading to increased expression of LXR-target genes. Thus, in *Pla2g10^−/−^* mice, elevated expression of the ATB-binding cassette (ABC) transporters ABCA1 and ABCG1 led to increased cholesterol efflux by macrophages [43], that of the steroidogenesis acute regulatory protein StAR resulted in increased corticosterone production by adrenal cells [44], and that of PPARγ (peroxisome proliferator-activated receptor γ) facilitated adipogenesis and adiposity [45]. On the contrary, *Pla2g10^−/−^* mice maintained on a chow diet over one year gradually lost body weight, most likely because dietary phospholipid digestion and thereby lipid absorption in the gastrointestinal tract was perturbed [38]. Collectively, these observations have highlighted a novel role of sPLA_2_-X in the regulation of metabolic states.

Finally, sPLA_2_-X is abundantly expressed in testicular spermatigenic cells and is released from the acrosome of capacitative (activated) sperm. *Pla2g10^−/−^* spermatozoa displayed reduced acrosome reaction and thereby reduced fertility, and this defect could be restored by LPC, a potential sPLA_2_-X-generated lipid product [32,38]. sPLA_2_-X is also expressed in peripheral neurons such as dorsal ganglion (DRG) neurons, and DRG from *Pla2g10^−/−^* mice showed reduced, whereas that from *Pla2g10*-Tg mice showed increased, *ex vivo* neuritogenesis [38]. Probably because of the altered neuritogenesis, pain nociception in the acetic acid writhing test was partially ameliorated in *Pla2g10^−/−^* mice, whereas it was augmented in *Pla2g10*-Tg mice, compared with that in littermate control mice [38].

### 2.3. Group III sPLA_2_ (sPLA_2_-III)

sPLA_2_-III is the only enzyme belonging to the group III collection. It is an unusually large protein (55 kDa) among the sPLA_2_ family and consists of three domains, in which a central sPLA_2_ domain displaying all the features of group III bee venom sPLA_2_, including 10 cysteines and the key residues of the Ca^2+^ loop and catalytic site, is flanked by large and unique N- and C-terminal region [46]. sPLA_2_-III is processed to a sPLA_2_ domain-only form (devoid of the N- and C-terminal domains), which is sufficient for its catalytic function [47,48]. sPLA_2_-III undergoes N-glycosylation and can hydrolyze PC and PE equally and augment arachidonate release from cell membranes more efficiently than sPLA_2_-IIA, and less efficiently than sPLA_2_-X and sPLA_2_-V. sPLA_2_-III is immunohistochemically detected in the vascular endothelium of various tissues, peripheral and central nervous systems, male reproductive tracts, and several types of cancer [48,49]. Implantation of sPLA_2_-III-transfected colorectal adenocarcinoma cells into nude mice promotes the growth of tumor xenografts [48]. Expression profiling of the full set of sPLA_2_s in human colon suggests that sPLA_2_-III might be a good candidate as a novel biomarker for colon cancers [50]. In the central nervous system, *Pla2g3* mRNA is localized in DRG neurons in mice, and overexpression of human sPLA_2_-III in cultured neuronal cells facilitates neurite outgrowth and survival in correlation with the production of LPC, whereas knockdown of endogenous sPLA_2_-III by siRNA partially suppresses these processes [49].

To address the potential *in vivo* action of sPLA_2_-III, we produced transgenic mice overexpressing this enzyme in the whole body (*Pla2g3*-Tg). Unlike *Pla2g5*-Tg mice, which die shortly after birth due to a lung disorder resulting from aberrant hydrolysis of the lung surfactant phospholipids (see above), *Pla2g3*-Tg mice showed no respiratory disorder, and lung surfactant phospholipids did not show appreciable difference between control and *Pla2g3*-Tg mice [51]. Furthermore, although *Pla2g10-*Tg mice show alopecia (see above), *Pla2g3*-Tg mice had normal pelage hairs up to nine months of age. Later on, however, *Pla2g3*-Tg mice spontaneously developed inflammation such as dermatitis, lymphocytic sialadenitis and splenomegaly [51]. The dermatitis was accompanied by hyperkeratosis, acanthosis, parakeratosis, erosion, ulcer, neutrophil infiltration, and increased production of proinflammatory cytokines, chemokines and prostaglandin E_2_ (PGE_2_). It is thus likely that overexpression of sPLA_2_-III facilitates the production of pro-inflammatory lipid mediators in the whole body, leading to systemic inflammation.

To look for potential substrates for sPLA_2_-III in *Pla2g3*-Tg mice, lipids extracted from splenocytes of aged *Pla2g3*-Tg and littermate control mice were subjected to ESI-MS analysis. Several PC molecular species were detected in splenocytes of wild-type (WT) mice, and their composition did not differ appreciably from those of *Pla2g3*-Tg mice (Figure 3a, *Upper*). However, a notable difference that could account for the PLA_2_-mediated lipolysis was seen in PS; of the detectable PS molecular species, PS with C18:0–18:1 (*m/z* = 790.6) were ∼50% less in *Pla2g3*-Tg mice than in control mice (Figure 3a, *Lower*). These results suggest that, in splenocyte membranes, PS with C18:0–18:1 may represent a major target substrate of sPLA_2_-III. Since PS is mainly present in the inner leaflet of the plasma membrane of live cells and exposed on apoptotic cell surfaces [52,53], extracellular sPLA_2_-III might preferentially hydrolyze PS with C18:0–18:1 on apoptotic cells and thereby modulate the life-span of inflammatory cells. In support of this idea, susceptibility of cell membranes to sPLA_2_s increases in apoptotic cells [54].

As in the case of sPLA_2_-V and -X, sPLA_2_-III can potently hydrolyze phospholipids in plasma lipoprtein particles [55]. Indeed, the decreased level of plasma lipoproteins, HDL in particular, was obvious in *Pla2g3*-Tg mice in comparison with WT mice (Figure 3b), suggesting HDL hydrolysis by overexpressed sPLA_2_-III. LDL treated with sPLA_2_-III *in vitro* was pro-atherogenic, promoting foam cell formation from macrophages. When *Pla2g3*-Tg mice that had been crossed with *ApoE^−/−^* mice (*Pla2g3^tg^/ApoE^−/−^*) were fed a high-cholesterol diet, lipid accumulation in the aortic walls was markedly increased as compared with replicate *ApoE^−/−^* mice (Figure 3c). Immunohistochemistry and *in situ* hybridization revealed the presence of sPLA_2_-III in human atherosclerotic plaques, particularly in macrophages and smooth muscle cells [55,56]. These results suggest that sPLA_2_-III may have a role in acceleration of atherosclerosis development [55].

sPLA_2_-III is expressed in the testis and epididymis, and in the latter tissue the mature form of sPLA_2_-III is secreted from the proximal epididymal epithelium into the lumen [57]. We have recently succeeded in generating *Pla2g3^−/−^* mice and found that they displayed male infertility [57]. Although testicular spermatogenesis in *Pla2g3^−/−^* mice was grossly normal, spermatozoa from the cauda (tail) epididymidis displayed hypomotility, and their ability to fertilize intact eggs was markedly impaired. Epididymal spermatozoa in *Pla2g3^−/−^* mice had aberrant acrosomal structures and flagella with abnormal axonemes. These results revealed an unexplored role of this atypical sPLA_2_ in epididymal lipid homeostasis, whose perturbation led to sperm dysfunction.

After the complex differentiation process of male germ cells, spermatozoa exit the seminiferous tubules of the testis through the efferent ducts toward the epididymis. During their transit from the caput (head) to the cauda (tail) epididymidis, sperm cells undergo significant morphological and biochemical modifications, which lead to acquisition of their forward motility and ability to recognize and fertilize oocytes [58]. Unique to mammalian sperm cells is the abundance of phospholipid species with C22-PUFAs, particularly docosahexaenoic acid (DHA) and docosapentaenoic acid (DPA), whose proportion in membrane phospholipids appears to correlate with sperm maturity, motility and fertility [59–62]. The percentage of DHA relative to total fatty acids is correlated with the normal morphology of sperm cells [61], and sperm from subfertile men with low sperm motility or counts contain a percentage of DHA lower than that from normal men [63]. Sperm maturation involves the remodeling of membrane phospholipids toward the acquisition of motility and fertility during sperm migration through the epididymis. Indeed, the increase in C22-PUFAs such as DHA and DPA and the reciprocal decrease in arachidonic acid (C20:4) favor an increase in the unsaturation degree of fatty acids in mouse sperm membrane during epididymal transit [59], which could consequently contribute to increasing the mouse sperm membranous fluidity [64,65]. Interestingly, ESI-MS analysis of sperm membrane phospholipids revealed that, during epididymal transit, PC in WT sperm underwent a dramatic shift in its acyl groups from oleic, linoleic and arachidonic acids to DPA and DHA, whereas this membrane lipid remodeling was compromised in *Pla2g3^−/−^* sperm [57]. Accordingly, cauda epididymal spermatozoa in *Pla2g3^−/−^* mice had PC species containing more oleate and less DHA/DPA than did those in *Pla2g3^+/+^* mice, a finding that appears to be consistent with the aforementioned notion that sperm with higher DHA percentages have better motility and fertility. Thus, sPLA_2_-III may participate in the hydrolysis of PC with oleic, linoleic and arachidonic acids in the sperm membrane during epididymal transit and that this event may be followed by reacylation of LPC, a PLA_2_ reaction product, with DHA and DPA, leading to an increase of PC with DPA/DHA in mature spermatozoa. In the *Pla2g3^−/−^* epididymis, impairment of the deacylation step may eventually perturb the subsequent reconstitution of DPA/DHA in the sperm membrane, culminating in the asthenozoospermia phenotype.

We also found a notable change in the ESI-MS/MS profile of lipid mediators in the epididymis of *Pla2g3^−/−^* mice [57]. Thus, arachidonate/linoleate metabolites of the 12/15-lipoxygenase (LOX) and cytochrome P450 (CYP450) pathways, but not those of the cyclooxygenase (COX) and 5-LOX pathways, were substantially reduced in the epididymis of *Pla2g3^−/−^* mice compared with that of *Pla2g3^+/+^* mice (Figure 4a). Although the role of 12/15-LOX or CYP450 metabolites in male fertility has not yet been fully established, expression of 12/15-LOX in spermatogenic cells has led to the suggestion that it may participate in sperm maturation [62]. In this context, the possibility that certain 12/15-LOX- or CYP450-derived lipid mediator(s) may be at least partly responsible for the regulation of sperm maturation by sPLA_2_-III should be taken into account.

Additionally, sPLA_2_-III may also affect lipid transport between sperm and epididymal epithelial cells. Several lipoprotein components are secreted by epididymal epithelial cells [67] and associate with and dissociate from sperm membranes scheduled for endocytosis by epididymal principal cells [68]. Male fertility can be impaired to various degrees by inactivation of the genes involved in lipoprotein metabolism [69–71]. In fact, membrane transport by epididymosomes, a particular lipoprotein membrane particle emitted from caput epididymal principal cells into the lumen, is fundamental for the process of sperm cell maturation in the epididymis [59,72]. Our speculation that sPLA_2_-III may also affect this epididymal lipid transport is supported by the finding that, as assessed by ESI-MS, the epididymal fluid from *Pla2g3^−/−^* mice contained PC more abundantly than that from *Pla2g3^+/+^* mice (Figure 4b). Taken together, we conclude that sPLA_2_-III may regulate epididymal sperm maturation through (i) regulation of phospholipid remodeling in sperm membranes, (ii) production of 12/15-LOX and CYP450 metabolites, and (iii) modification of lipid transport between sperm and epididymal epithelial cells (Figure 4c).

### 2.4. Other sPLA_2_s: Classical and Novel Enzymes

Group IB pancreatic sPLA_2_ (sPLA_2_-IB) is synthesized in the pancreatic acinar cells, and after secretion into the pancreatic juice, an N-terminal heptapeptide of the inactive zymogen is cleaved by trypsin to yield an active enzyme in the duodenum [74]. The main role of sPLA_2_-IB is digestion of dietary and biliary phospholipids. Thus, perturbation of this process by gene disruption (*Pla2g1b^−/−^*) or pharmacological inhibition of sPLA_2_-IB led to protection from diet-induced obesity and insulin resistance due to decreased lipid digestion and absorption in the gut [75,76]. In agreement, the *PLA2G1B* gene resides within a locus for obesity susceptibility in humans [77].

Group IIA sPLA_2_ (sPLA_2_-IIA) is often referred to as an inflammatory sPLA_2_, since its expression is markedly induced during inflammation, cardiovascular diseases, and tissue damages [78]. When overexpressed, sPLA_2_-IIA is capable of augmenting arachidonic acid release in cytokine-stimulated cells, albeit more weakly than sPLA_2_-V, -X and -III [79]. Despite these facts, the contribution of sPLA_2_-IIA to inflammation has remained a subject of debate until recently, since a natural mutation of its gene in C57BL/6 and 129Sv mice [80] prevents the proper assessment of its functions by a classical gene targeting strategy. Intrinsic deficiency of sPLA_2_-IIA in these mouse strains is associated with increased incidence of intestinal polyposis and tumorigengesis [80], a phenotype that is reversed by transgenic expression of the *Pla2g2a* gene [81]. A recent study using *Pla2g2a*-deficient BALB/c mice as well as *Pla2g2a*-Tg mice has provided compelling evidence that the enzyme plays an exacerbating role in inflammatory arthritis [26]. The best-recognized physiologic function of sPLA_2_-IIA is the degradation of Gram-positive bacterial membrane, thereby providing the first line of antimicrobial defense of the host [82–85]. The serum level of sPLA_2_-IIA also shows correlation with the risk of cardiovascular diseases [86], and *Pla2g2a*-Tg mice fed an atherogenic diet developed atherosclerosis [87,88]. This effect is probably because sPLA_2_-mediated hydrolysis of LDL phospholipids leads to generation of small-dense, pro-atherogenic LDL particles that facilitate macrophage foam cell formation, even though the hydrolytic activity of sPLA_2_-IIA toward lipoportein particles is much weaker than that of sPLA_2_-V, -X and -III. *Pla2g2a*-Tg mice also displayed permanent alopecia and were susceptible to carcinogen-induced skin tumorigenesis [39,40].

The roles of other group II subfamily sPLA_2_ isoforms remain elusive, since knockout or transgenic mice for these enzymes have not yet been reported. sPLA_2_-IIC is expressed in rodent testis, but not in humans [89]. sPLA_2_-IID is structurally most similar to sPLA_2_-IIA, and its transcript is constitutively detected in the lymphoid organs [90]. This enzyme may have immuno-suppressive functions, since it is expressed in regulatory T cells and its fusion protein has the ability to suppress inflammatory bowel disease and experimental autoimmune encephalomyelitis in mice [91]. sPLA_2_-IIE, another group IIA-related enzyme, is expressed constitutively in several tissues at low levels and has a lower catalytic activity than other group II sPLA_2_s [92]. sPLA_2_-IIF possesses a unique 30-amino acid C-terminal extension that contains an additional Cys residue, which might contribute to formation of a homodimer or a heterodimer with a second protein [93,94]. This enzyme is expressed most abundantly in the skin [100].

Lastly, group XII sPLA_2_s (sPLA_2_-XIIA and -XIIB) represent a unique collection of the sPLA_2_ family. sPLA_2_-XIIA has the central catalytic domain with a His/Asp catalytic dyad, yet the location of Cys residues outside the catalytic domain is rather distinct from that of other sPLA_2_s [95]. High expression of this enzyme is found in many tissues, although its enzymatic activity is very weak. A study using *Xenopus* suggests the role of this enzyme in early neuronal development [96]. sPLA_2_-XIIB is structurally related to sPLA_2_-XIIA and is expressed in liver and intestine [97]. A recent study has demonstrated that the transcription of *Pla2g12b* was regulated by the transcription factor HNF-4α and its co-activator PGC-1α, and deletion of the *Pla2g12b* gene resulted in increased fat accumulation in the liver leading to steatohepatitis, a phenotype similar to that seen in *Hnf4a^−/−^* mice [98]. The aberrant fat accumulation in *Pla2g12b^−/−^* liver was ascribed to impaired hepatic secretion of VLDL. However, because sPLA_2_-XIIB lacks the catalytic activity since the catalytic center His is replaced with Leu [97], the molecular mechanism whereby this sPLA_2_ isoform regulates VLDL secretion remains unknown.

## 3. Conclusions

During the past decade, the biological functions of several sPLA_2_s and their target substrates have been clarified by studies using transgenic and knockout mice in combination with lipidomics. Nevertheless, full understanding of the biological roles of all sPLA_2_ isoforms is still a challenging area of research. The control of particular sPLA_2_s, alone or in combination of multiple isoforms, should have advantages over the inhibition of selective lipid metabolic pathways in the treatment of various diseases. Interestingly, the pan-sPLA_2_ inhibitor A-002 (varespladib), which inhibits the conventional class of sPLA_2_s, can markedly reduce the atherosclerotic lesion area in experimental animals and even in humans in early-phase clinical studies [99]. This fact points to the sPLA_2_ family as a potential therapeutic target for atherosclerosis, and probably other diseases in which one or more sPLA_2_s are involved, such as asthma, arthritis, and metabolic syndrome.

## Figures and Tables

**Figure 1.** *Pla2g5*-Tg mice display fatal respiratory failure due to lung surfactant destruction**. (a** and **b)** ESI-MS of surfactant PC (**a**) and PG (**b**) from *Pla2g5*-Tg mice (*right*) and WT mice (*left*); Molecular peaks shown in red, such as PC32:0 (16:0–16:0) and PC32:1 (16:0–16:1) (**a**) as well as PG32:0 (16:0–16:0), PG34:1 (16:0–18:1), PG36:4 (16:0–20:4) and PG38:6 (16:0–22:6); (**b**) were dramatically reduced in *Pla2g5*-Tg mice compared with WT mice. IS, internal standard; **(c)** RT-PCR of sPLA_2_-V mRNA in cultured human bronchial epithelial cells with or without stimulation for 12 h with pro-inflammatory cytokines. sPLA_2_-V was induced by IL-1β or TNFα but not by IFNγ; (**d**) A schematic model of the role of sPLA_2_-V in lung surfactant hydrolysis. sPLA_2_-V is secreted from bronchial epithelial cells and alveolar macrophages stimulated with pro-inflammatory cytokines, and aberrant hydrolysis of surfactant PC and PG by sPLA_2_-V leads to airway injury. For details, see [8].

**Figure 2.** *Pla2g10*-Tg mice display alopecia during the postnatal hair cycle. (**a**) *Pla2g10*-Tg mice displayed temporary alopecia during 2–3 wk after birth, a period of the postnatal hair cycle; (**b**) Histology of 3-wk-old *Pla2g10*-Tg mice, in comparison with that of WT mice, revealed hair follicle distortion as well as epidermal hyperplasia, sebaceous gland enlargement, and cyst formation; (**c**) ESI-MS of skin phospholipids indicated that PE molecular species with PUFA (arachidonic acid (C20:4) and docosahexaenoic acid (C22:6)), but not PC, was markedly decreased in *Pla2g10*-Tg mice compared with WT mice; (**d**) A schematic model of the sPLA_2_-X action in the skin. sPLA_2_-X is converted by certain skin proteases to its active form, which then hydrolyzes PE in skin membranes to liberate PUFA that is further metabolized to skin-acting eicosanoids; (**e**) Endogenous sPLA_2_-X is localized in the ORS of hair follicles (shown in red). ORS, outer root sheath; IRS, inner root sheath. For details, see [38].

**Figure 3.** *Pla2g3*-Tg mice display systemic inflammatory and atherosclerotic phenotypes**. (a)** ESI-MS of PC and PS in splenocytes from *Pla2g3*-Tg (III-Tg) and wild-type (WT) mice. Major peaks are indicated by arrows. Peaks altered in III-Tg mice relative to WT mice are shown in red. SM, sphingomyelin; **(b)** HPLC profile of plasma lipoproteins in III-Tg and WT mice; **(c)** Increased atherosclerosis in III-Tg mice on the *ApoE^−/−^* background (male, 24-wk-old). Atheroslcerotic lesions were visualized by oil red O staining. Areas positive for the staining were quantified. For details, see [51,55].

**Figure 4.** *Pla2g3^−/−^* mice have multiple defects in epididymal sperm maturation. **(a)** Altered eicosanoid levels in *Pla2g3^−/−^* mice. The levels of individual eicosanoids in the epididymis were determined by LC-ESI-MS/MS. sPLA_2_-III is selectively coupled with 12/15-LOX and CYP450 pathways; **(b)** Unusual accumulation of PC molecular species in the epididymal fluids from *Pla2g3^−/−^* mice relative to *Pla2g3^+/+^* mice, as assessed by ESI-MS; (**c**) The roles of sPLA_2_-III in epididymal sperm maturation are summarized. For details, see [57].

**Table 1.** *In vitro* actions of sPLA_2_s on various membranes.

**sPLA_2_s**		**resting cell membrane**	**activated cell membrane**	**lipoprotein (PC)**	**surfactant (PC)**	**Gram-positive bacteria**	**Gram-negative bacteria**
conventional sPLA_2_s	IB	weak	moderate	weak	weak	none	none
	IIA	none	moderate	weak	weak	very high	weak*
	IID	none	weak	n.d.	weak	high	none
	IIE	none	weak	n.d.	n.d.	moderate	none
	IIF	moderate	moderate	moderate	n.d.	none	none
	V	high	very high	very high	very high	high	none
	X	very high	very high	very high	high	moderate	none
atypical sPLA_2_s	III	moderate	moderate	high	n.d.	n.d.	none
	XIIA	none	none	n.d.	n.d.	high	moderate

n.d.; not determined. sPLA_2_-IIC is not included since it is a pseudogene in human.

* sPLA_2_-IIA kills Gram-negative bacteria only in the presence of bacterial permeability-increasing protein.

For details, please see refs [30,31,41,47,55,79,85,94].

## Abbreviations:

PLA_2_: phospholipase A_2_;
sPLA_2_: secreted PLA_2_;
cPLA_2_: cytosolic PLA_2_;
iPLA_2_: Ca^2+^-independent PLA_2_;
Tg: transgenic;
ARDS: acute respiratory distress syndrome;
BALF: bronchoalveolar fluid;
LPS: lipopolysaccharide;
ESI-MS: electrospray ionization mass spectrometry;
PC: phosphatidylcholine;
LPC: lysophosphatidylcholine;
PG: phosphatidylglycerol;
PE: phosphatidylethanolamine;
PS: phosphatidylserine;
LDL: low-density lipoprotein;
HDL: high-density lipoprotein;
VLDL: very low-density lipoprotein;
ABC: ATP-binding cassette;
PGD_2_: prostaglandin D_2_;
PGE_2_: prostaglandin E_2_;
LTB_4_: leukotriene B_4_;
PUFA: polyunsaturated fatty acid;
DHA: docosahexaenoic acid;
DPA: docosapentaenoic acid;
LXR: liver X receptor;
PPAR: peroxisome proliferator-activated receptor;
StAR: steroidogenic acute regulatory protein;
DRG: dorsal root ganglion;
COX: cyclooxygenase;
LOX: lipoxygenase;
CYP450: cytochrome P450;
HPLC: high performance liquid chromatography;
WT: wild-type.
